The article "Intrahemispheric EEG: A New Perspective for Quantitative EEG Assessment in Poststroke Individuals" was published in 2021. Journal: Neural Plast.

# Intrahemispheric EEG: A New Perspective for Quantitative EEG Assessment in Poststroke Individuals

**DOI:** 10.1155/2021/5664647

**Published:** 2021-09-21

**Authors:** Rodrigo Brito, Adriana Baltar, Marina Berenguer-Rocha, Lívia Shirahige, Sérgio Rocha, André Fonseca, Daniele Piscitelli, Kátia Monte-Silva

**Affiliations:** ^1^Applied Neuroscience Laboratory, Department of Physical Therapy, Universidade Federal de Pernambuco, Recife, Pernambuco, Brazil; ^2^NAPeN Network (Núcleo de Assistência e Pesquisa em Neuromodulação), Brazil; ^3^Center of Mathematics, Computation and Cognition, Universidade Federal do ABC, Sao Paulo, Brazil; ^4^School of Medicine and Surgery, University of Milano Bicocca, Milano, Italy; ^5^School of Physical and Occupational Therapy, McGill University, Montreal, Canada

## Abstract

The ratio between slower and faster frequencies of brain activity may change after stroke. However, few studies have used quantitative electroencephalography (qEEG) index of ratios between slower and faster frequencies such as the delta/alpha ratio (DAR) and the power ratio index (PRI; delta + theta/alpha + beta) for investigating the difference between the affected and unaffected hemisphere poststroke. Here, we proposed a new perspective for analyzing DAR and PRI within each hemisphere and investigated the motor impairment-related interhemispheric frequency oscillations. Forty-seven poststroke subjects and twelve healthy controls were included in the study. Severity of upper limb motor impairment was classified according to the Fugl–Meyer assessment in mild/moderate (*n* = 25) and severe (*n* = 22). The qEEG indexes (PRI and DAR) were computed for each hemisphere (intrahemispheric index) and for both hemispheres (cerebral index). Considering the cerebral index (DAR and PRI), our results showed a slowing in brain activity in poststroke patients when compared to healthy controls. Only the intrahemispheric PRI index was able to find significant interhemispheric differences of frequency oscillations. Despite being unable to detect interhemispheric differences, the DAR index seems to be more sensitive to detect motor impairment-related frequency oscillations. The intrahemispheric PRI index may provide insights into therapeutic approaches for interhemispheric asymmetry after stroke.

## 1. Introduction

Stroke is one of the leading causes of adult disability worldwide [1]. Following a stroke, an imbalance in the interhemispheric cortical interaction may be established [2]. The ability to perform skilled limb movements requires a dynamic interaction between the hemispheres. Maladaptive functioning of this interhemispheric interaction and consequently changes in hemisphere neural activity after stroke are thought to be factors underlying motor impairments and the poorest motor recovery in these patients [3–5].

The article "Intrahemispheric EEG: A New Perspective for Quantitative EEG Assessment in Poststroke Individuals" was published in 2021. Journal: Neural Plast.

The abnormal interhemispheric interaction after a brain injury has been mainly investigated by functional magnetic resonance imaging (fMRI), positron emission tomography (PET), and transcranial magnetic stimulation (TMS) [5, 6]. The quantitative electroencephalography (qEEG) may also be a reliable instrument for detecting alterations of interhemispheric interaction poststroke. The presence of low-frequency oscillations (delta and theta rhythm) in the EEG signal is linked to the decline in neuronal integrity [7, 8], whereas the presence of fast-frequency oscillations (alpha, beta, and gamma rhythm) after stroke is associated with the motor recovery and functional outcome following stroke [7, 9]. Thus, the qEEG index of ratio between slower and faster frequencies such as the delta/alpha ratio (DAR) [10], the power ratio index (PRI; delta + theta/alpha + beta) [11, 12], and the theta/beta ratio (TBR) [13, 14] has been largely employed in stroke studies [10, 13, 15–19].

However, to the best of our knowledge, few studies have used PRI and DAR indexes for investigating the difference between affected and unaffected hemisphere in poststroke subjects. In a recent study, Fanciullacci et al. (2017) did not find any significant interhemispheric difference for DAR in subacute poststroke individuals with cortical-subcortical and subcortical lesions. Moreover, Fanciullacci et al. [18] did not consider motor impairment severity, while recent findings using TMS suggested that cortical activity changes within both hemispheres are strongly associated with motor impairments [20].

Our matched controlled study proposed a new perspective for the analysis of these qEEG indexes within each hemisphere. We hypothesized that ratios between slower and faster frequencies in each hemisphere would be more appropriate to study neural activity changes for considering the interhemispheric differences after stroke. Moreover, we expected that such interhemispheric differences of DAR and PRI after stroke might critically depend on motor impairments.

## 2. Methods

### 2.1. Participants

Forty-seven poststroke patients were recruited from local rehabilitation clinics. These patients had mild/moderate (25; 52% males; mean age: 59.6) and severe (22; 45.5% males; mean age: 58.2) motor impairment based on the upper limb section of the Fugl–Meyer assessment [21]. It included patients with upper limb hemiparesis resulting from ischemic or hemorrhagic stroke (>3 months) aged from 18 to 75 years old. We excluded patients with cognitive impairment (<18 in the mini mental state examination (MMSE)) or with any psychiatric disorder. As a control study, self-reported healthy volunteers aged and sex-matched with the patients were also included in the study. This study was reviewed and approved by the local human ethical committee. All patients and healthy controls signed the informed consent before participating in the study. Clinical sociodemographic characteristics were collected. Handedness was self-reported.

The article "Intrahemispheric EEG: A New Perspective for Quantitative EEG Assessment in Poststroke Individuals" was published in 2021. Journal: Neural Plast.

### 2.2. Motor Impairment Severity

The upper limb section of the Fugl–Meyer assessment (UL-FMA) with a maximum score of 66 [21] was applied to evaluate the level of motor impairment. Poststroke patients were classified: with mild/moderate (>19 ± 2 points in UL-FMA) and with severe motor impairment (<19 ± 2 points) according to the classification described by Woodbury et al. [22].

### 2.3. EEG Data Acquisition and Processing

EEG was recorded for 60 seconds in an isolated room with volunteers with eyes opened and seated in a comfortable armchair, as recommended by the American Clinical Neurophysiology Society Guideline [23, 24]. EEG was recorded using a digital EEG equipment (Neuron-Spectrum/Neurosoft, Russia) with nine Ag/AgCl scalp electrodes placed at F3, C3, P3, Fz, Cz, Pz, F4, C4, and P4 and the reference electrodes at A1 and A2 according to the international 10/20 system at a sampling frequency of 500 Hz. The electrode impedances were kept well below 15 k*Ω*. The signal was filtered with a bandpass (0.5–100 Hz) and a notch filter of 60 Hz.

Offline signal processing was performed by the toolbox EEGLab in the MATLAB® R2014a for Windows. EEG data file was segmented into 30 data points. The artifact analysis was performed in the continuous data by the independent component analysis (ICA) with the RUNICA algorithm. The ICA may be used to remove artifacts embedded in the data (muscle, eye blinks, or eye movement) without removing the affected data position. Following the identification of the artifacts, the rejection was performed by the Multiple Artifact Rejection Algorithm (MARA), considering a cutoff of 50% [25]. Then, the spectral power density (PSD) was computed for each electrode using the Welch estimator, through an approximation of the edge over the Hanning window [26]. The absolute power was calculated for delta (*δ*) (0.5 to ≤4 Hz), theta (*θ*) (>4 to ≤8 Hz), alpha (*α*) (>8 to ≤13 Hz), beta (*β*) (>13 to ≤30 Hz), and gamma (*γ*) (<30 *a* ≤ 45 Hz) [27]. Moreover, the relative band power was calculated by dividing each band's absolute band power with the total power in 0.5-45 Hz. The relative power at each electrode was averaged to obtain global relative power and this global relative power was used to calculate power ratio index (PRI), delta to alpha ratio (DAR), and theta to beta ratio (TBR). PRI was calculated as PRI = (*rδ* + *rθ*)/(*rα* + *rβ*) [11]. DAR was calculated as DAR = *rδ*/*rα* [10]. TBR was calculated as TBR = *rθ*/*rβ* [13].

The article "Intrahemispheric EEG: A New Perspective for Quantitative EEG Assessment in Poststroke Individuals" was published in 2021. Journal: Neural Plast.

The qEEG index (PRI and DAR) was computed for each hemisphere (intrahemispheric index) and for both hemispheres (cerebral index). The intrahemispheric index was defined as the mean of the global relative power over electrodes within each hemisphere (left side: F3, C3, and P3; right side: F4, C4, and P4). The cerebral index was defined as the mean of the global relative power over all nine electrodes (F3, C3, P3, Fz, Cz, Pz, F4, C4, and P4).

### 2.4. Data Analysis

Kolmogorov-Smirnov was performed to assess the data normality. First, the independent sample *t*-test was used to compare the cerebral index between poststroke patients and healthy volunteers. One-way ANOVA repeated measure analysis for each population separately (poststroke and healthy volunteers) was performed for the intragroup comparison among each intrahemispheric index and cerebral index. For poststroke patients, a two-way ANOVA repeated measure with intrahemispheric/cerebral index (affected hemispheric index, unaffected hemispheric index, and cerebral index) as within factor and motor impairment (mild/moderate and severe) as between factors was performed. When necessary, post hoc analysis was performed using *t*-test. For multiple comparisons, Bonferroni's correction was applied. Mauchly's sphericity was checked, and Greenhouse-Geisser correction was performed when necessary. For all analysis, the observed power of statistical (*η*^2^) analysis was calculated; also, the *t*-test Cohen's D (*d*) was reported. Statistical analysis was performed using SPSS (Statistical Package for the Social Sciences) software 20.0 for Windows, adopting a significance level (*p*) of 0.05.

## 3. Results

Fifty-six poststroke patients and fourteen healthy volunteers were assessed. Nine poststroke patients and two healthy volunteers had the data missing for EEG acquisition errors. Thus, forty-seven poststroke and twelve healthy volunteers had the data analyzed.  Figure 1 shows the flowchart of the volunteers in the study.  Table 1 depicts the demographic and clinical characteristics of the participants.

### 3.1. Power Ratio Index

Considering the cerebral index, the independent sample *t*-test revealed a slowing in brain activity in poststroke patients when compared to healthy volunteers (poststroke: 2.71 ± 0.51; healthy: 2.09 ± 0.71; *d* = 1.00; *t* = 3.41; *p* = 0.001).

The one-way ANOVA showed a significant effect of intrahemispheric/cerebral index for the poststroke patients (*F*_(1.06,48.6)_ = 10.74; *p* = 0.02; *η*^2^ = 0.91), but not for healthy volunteers (*F*_(1.01, 12.1)_ = 0.38; *p* = 0.57; *η*^2^ = 0.09). The post hoc analysis revealed an increased intrahemispheric PRI index in the affected hemisphere when compared to the unaffected intrahemispheric (affected hemisphere: 2.75 ± 0.54; unaffected hemisphere: 2.63 ± 0.47; *d* = 0.23; *t* = −3.26; *p* = 0.002) and cerebral index (cerebral index: 2.71 ± 0.51; *d* = 0.07; *t* = 2.20; *p* = 0.03). A decreased intrahemispheric PRI index in the unaffected hemisphere was found when compared to cerebral index (unaffected hemisphere: 2.62 ± 0.47; cerebral index: 2.71 ± 0.51; *d* = 0.18; *t* = −3.91; *p* < 0.001).

The article "Intrahemispheric EEG: A New Perspective for Quantitative EEG Assessment in Poststroke Individuals" was published in 2021. Journal: Neural Plast.

The two-way ANOVA showed a significant main effect for intrahemispheric/cerebral index (*F*_(1.06, 47.8)_ = 12.65; *p* = 0.001; *η*^2^ = 0.95) and for interaction between the two main factors (*F*_(1.06, 47.8)_ = 5.14; *p* = 0.026; *η*^2^ = 0.62), but not for motor impairment factor (*F*_(1, 45)_ = 2.72; *p* = 0.11; *η*^2^ = 0.36). In contrast to healthy controls (non-domH: 2.08 ± 0.70; domH: 2.11 ± 0.67; *d* = 0.04; *t* = 0.64; *p* = 0.54) and poststroke patients with mild/moderate motor impairment (mild/moderate-affected hemisphere: 2.60 ± 0.41; mild/moderate-unaffected hemisphere: 2.56 ± 0.41; *d* = 0.09; *t* = −1.62; *p* = 0.12), the post hoc analysis revealed a significant difference between intrahemispheric PRI index of the affected and nonaffected hemisphere in the patients with severe motor impairment (severe-affected hemisphere: 2.91 ± 0.62; severe-unaffected hemisphere: 2.70 ± 0.51; *d* = 0.36; *t* = −3.00; *p* = 0.007). All intrahemispheric PRI index differed to the cerebral index, except for the affected hemisphere of poststroke patients with mild/moderate motor impairment (mild/moderate cerebral index: 2.60 ± 0.41; severe cerebral index: 2.83 ± 0.59; *d* = 0.45; *t* = −3.91; *p* < 0.001).  Table 2 shows the intrahemispheric and cerebral power ratio index (PRI) in poststroke patients with upper limb mild/moderate and severe motor impairment and healthy subjects.

### 3.2. Delta to Alpha Ratio

Similar to cerebral PRI index, the independent sample *t*-test revealed a statistical slowing in brain activity, as revealed by increased DAR index, in poststroke patients when compared to healthy controls (poststroke: 2.20 ± 0.36; healthy: 1.79 ± 0.50; *d* = 0.94; *t* = 3.28; *p* = 0.02).  Table 3 shows the DAR in poststroke and healthy individuals.

The one-way ANOVA showed no significant effect of intrahemispheric/cerebral index for the poststroke patients (*F*_(1.69,77.9)_ = 0.22; *p* = 0.80; *η*^2^ = 0.08) and for healthy controls (*F*_(1.07,11.8)_ = 0.19; *p* = 0.83; *η*^2^ = 0.08).

The article "Intrahemispheric EEG: A New Perspective for Quantitative EEG Assessment in Poststroke Individuals" was published in 2021. Journal: Neural Plast.

The two-way ANOVA showed a significant effect only for motor impairment factor (*F*_(1, 45)_ = 13.11; *p* = 0.01; *η*^2^ = 0.94). The post hoc test revealed increased DAR index for poststroke patients with severe motor impairment when compared to the mild/moderate motor impairment for intrahemispheric index (mild/moderate-affected hemisphere: 2.06 ± 0.29; severe-affected hemisphere: 2.41 ± 0.26; *d* = 1.27; *t* = −4.30; *p* < 0.001; mild/moderate-unaffected hemisphere: 2.05 ± 0.32; severe-unaffected hemisphere: 2.36 ± 0.42; *d* = 0.83; *t* = −2.90; *p* = 0.006) and for cerebral index (mild/moderate: 2.07 ± 0.31; severe: 2.35 ± 0.36; *d* = 0.83; *t* = −2.87; *p* = 0.006).

### 3.3. Theta to Beta Ratio

Even as PRI and DAR, the independent sample *t*-test revealed an increased TBR index meaning a statistical slowing in brain activity in poststroke patients when compared to healthy controls (poststroke: 5.07 ± 2.18; healthy: 2.09 ± 0.71; *d* = 1.83; *t* = 7.85; *p* < 0.01).  Table 4 shows the TBR in poststroke and healthy controls.

Similar to the PRI index, the one-way ANOVA showed a statistical difference for intrahemispheric/cerebral index for the poststroke patients (*F*_(1.04,47.99)_ = 5.60; *p* = 0.02; *η*^2^ = 0.65) and no differences for healthy volunteers (*F*_(1.09,12.08)_ = 0.38; *p* = 0.56; *η*^2^ = 0.09). The post hoc analysis showed an increased intrahemispheric TBR index in the affected hemisphere when compared to the unaffected intrahemispheric (affected hemisphere: 5.39 ± 2.44; unaffected hemisphere: 4.85 ± 2.09; *d* = 0.23; *t* = −2.38; *p* = 0.02) and cerebral index (cerebral index: 5.07 ± 2.18; *d* = 0.13; *t* = 2.51; *p* = 0.01). In addition, a decreased intrahemispheric TBR index in the unaffected hemisphere was found when compared to cerebral index (*d* = 0.10; *t* = −2.04; *p* = 0.04).

According to the motor impairment analysis, the two-way ANOVA showed a significant main effect for intrahemispheric/cerebral index (*F*_(1.04, 47.07)_ = 6.32; *p* = 0.01; *η*^2^ = 0.70). However, no interaction was revealed between the two main factors (*F*_(1.04, 47.07)_ = 2.80; *p* = 0.09; *η*^2^ = 0.38) and for motor impairment factor (*F*_(1, 45)_ = 3.48; *p* = 0.06; *η*^2^ = 0.44). In addition, the post hoc analysis revealed a significant difference between intrahemispheric TBR index only for the severe motor impairment poststroke patients in the affected and unaffected hemisphere (severe-affected hemisphere: 6.21 ± 2.70; severe-unaffected hemisphere: 5.27 ± 2.37; *d* = 0.37; *t* = −2.35; *p* = 0.02), affected hemisphere and cerebral index (severe cerebral index: 5.66 ± 2.49; *d* = 0.21; *t* = 2.33; *p* = 0.03), and unaffected hemisphere and cerebral index (*d* = 0.16; *t* = −2.17; *p* = 0.04).

The article "Intrahemispheric EEG: A New Perspective for Quantitative EEG Assessment in Poststroke Individuals" was published in 2021. Journal: Neural Plast.

## 4. Discussion

As expected, we found a slowing brain electrical activity of poststroke patients. The presence of low-frequency oscillations (delta and theta) has been associated with brain injuries, as in our poststroke patients [28, 29].

A previous study has investigated the PSD in acute poststroke, showing a higher delta power in poststroke patients when compared to healthy volunteers [10, 30] and in the affected hemisphere of subcortical poststroke patients [18]. The delta oscillations originate in neurons in the thalamus and in deep cortical layers, which may reflect hyperpolarization and inhibition of cortical neurons, resulting in a decrease in neural activity [31]. In addition, it is expected in the poststroke patients, a suppression of high frequency alpha and beta band rhythms [32], since the presence of these rhythms is functionally related to the sensorimotor system, which is activated through motor preparation or execution [33].

In our study, we found an increased intrahemispheric PRI and TBR index in the affected hemisphere when compared to unaffected intrahemispheric and cerebral index and a decreased intrahemispheric PRI and TBR index in the unaffected hemisphere when compared to cerebral index. An increase in these indexes in a specific brain hemisphere supports our hypothesis that the qEEG index for the poststroke patients should be assessed to separate the affected and unaffected hemispheres. PRI seems to be a sensitive index to detect interhemispheric changes in cortical activity.

These findings were in line with previous studies that measure poststroke cerebral and interhemispheric activity by fMRI or TMS [34, 35]. The interhemispheric activity has been used as a surrogate outcome and prognostic factor to predict and monitor stroke progression [15, 34]. In this way, this imbalance could represent the worst prognosis as suggested by Min et al. (2019), which demonstrated slow PSD in the affected hemisphere, while the unaffected hemisphere has a higher PSD.

In contrast to the PRI and TBR indexes, the DAR analysis did not show a difference between the affected and unaffected hemispheres (intrahemispheric DAR index) or in comparison to the cerebral DAR index. Theta band is a potential predictive biomarker for cognitive impairment in patients with cerebral infarcts [36]. The TBR index is also a biomarker of brain processes involved in executive control processes [36], that is, the theta contribution can bring more and valuable information about the poststroke patient. The beta contribution in PRI measure is expected to be increased to determine a better motor recovery outcome (smaller PRI). Indeed, the increase of fast qEEG waves, especially beta rhythm, had been associated with motor recovery in poststroke [7, 9].

The article "Intrahemispheric EEG: A New Perspective for Quantitative EEG Assessment in Poststroke Individuals" was published in 2021. Journal: Neural Plast.

Another interesting result is related to the severity of motor impairment. The DAR seems to be a more sensitive index to assessing the severity of the motor impairment in poststroke patients than the PRI index. This trend could be seen for the affected and unaffected hemispheres of the interhemispheric index, as well as for the cerebral index. At the same time, the PRI had detected the difference only at the affected hemisphere. This finding supports the current literature that shows an association between DAR and clinical outcomes [29, 37]. The presence of alpha oscillation indicates neuronal survival [38] and indirectly reflects a decreased DAR. Some studies have demonstrated that the extension of area affected by the infarct is related to motor severity and recovery [39].

Some studies have claimed that an imbalance between interhemispheric connections is related to the severity of the sensorimotor impairment and to the motor recovery post cerebral infarct [2, 6, 20, 37].

Understanding the behavior of the affected and unaffected hemisphere and the severity of motor impairment of the poststroke patients can allow some interventions targeting the individual need, as through neurofeedback by brain-computer interface [14, 19, 40]. With the present study results, we would to suggest a neurofeedback aiming the increase of beta rhythm and decrease of delta for the reduction of the hemispheric PRI in the affected hemisphere.

The main limitation of this study was the limited number of channels in EEG acquisition. We used nine channels that were distributed to capture the cerebral activity of the right and left hemispheres. The extension and lesion location of the affected hemisphere were not controlled. Indeed, evidence suggests that EEG response can vary in patients with stroke depending on lesion [41].

## 5. Conclusion

The intrahemispheric PRI and TBR indexes are able to find significant interhemispheric differences of frequency oscillations. Despite being unable to detect interhemispheric differences, the DAR index seems to be more sensitive to detect motor impairment-related frequency oscillations. As PRI has the four more usable EEG frequency (delta, theta, alpha, and beta), the intrahemispheric PRI index could provide insights into a precise therapeutic approach through noninvasive brain stimulation or neurofeedback for interhemispheric asymmetry after stroke. These results point out a new perspective of analysis for the cerebral activity in poststroke patients, which could be used as a biomarker of motor recovery and/or as a prognostic measure. Additionally, DAR is the more sensitive index to assessing the severity of motor impairment. This information added to the analysis of each hemisphere's spectral power could guide some interventions as neurofeedback or noninvasive brain stimulations.

The article "Intrahemispheric EEG: A New Perspective for Quantitative EEG Assessment in Poststroke Individuals" was published in 2021. Journal: Neural Plast.

## Figures and Tables

**Figure 1:** Flowchart of the study.

**Table 1:** Demographic and clinical characteristics of participants.

	Poststroke patients		Healthy volunteers (*n* = 12)
	Mild/moderate motor impairment (*n* = 25)	Severe motor impairment (*n* = 22)	
Age, mean ± SD (years)	59.6 ± 8.4	58.2 ± 10.0	53.3 ± 6.3
Gender (%)			
Male	52%	45.5%	50%
Handedness (%)			
Right	88%	95.5%	91.7%
UL-FMA, mean ± SD (score)	38.7 ± 12.5	12.2 ± 4.0	—
Hemiparesis (%)			
Left	60%	63.6%	—
Time since stroke, mean ± SD (months)	38.3 ± 32.7	54.9 ± 40.4	—

SD: standard deviation; UL-FMA: upper limb Fugl–Meyer assessment.

**Table 2:** Intrahemispheric and cerebral power ratio index (PRI) in poststroke patients with upper limb mild/moderate and severe motor impairment and healthy subjects.

	Intrahemispheric index		Cerebral index	Within-group differences		
	Affected/non-domH	Unaffected/domH		Affected/non-domH vs. unaffected/domH	Affected/non-domH vs. cerebral index	Affected/domH vs. cerebral index
Healthy	2.08 ± 0.70	2.11 ± 0.67	2.10 ± 0.71	—	—	—
Poststroke patients	2.75 ± 0.54	2.63 ± 0.47	2.71 ± 0.51	*t* = −3.26; *p* = 0.002	*t* = 2.20; *p* = 0.03	*t* = −3.91; *p* < 0.001
Mild/moderate	2.60 ± 0.41	2.56 ± 0.41	2.60 ± 0.41	—	—	—
Severe	2.91 ± 0.62	2.70 ± 0.53	2.83 ± 0.59	*t* = −3.00; *p* = 0.007	—	—

non-domH: nondominant hemisphere; domH: dominant hemisphere. Data are mean ± SD. Significant post hoc test values for within-group differences are shown.

**Table 3:** Intrahemispheric and cerebral delta to alpha ratio (DAR) in poststroke patients with upper limb mild/moderate and severe motor impairment and healthy subjects.

	Intrahemispheric index		Cerebral index
	Affected/non-domH	Unaffected/domH	
Healthy	1.77 ± 0.49	1.79 ± 0.48	1.79 ± 0.50
Poststroke patients	2.22 ± 0.32	2.20 ± 0.40	2.20 ± 0.36
Mild/moderate	2.06 ± 0.29	2.05 ± 0.32	2.07 ± 0.31
Severe	2.41 ± 0.26	2.36 ± 0.42	2.35 ± 0.36

non-domH: nondominant hemisphere; domH: dominant hemisphere. Data are mean ± SD.

**Table 4:** Intrahemispheric and cerebral theta to beta ratio (TBR) in poststroke patients with upper limb mild/moderate and severe motor impairment and healthy subjects.

	Intrahemispheric index		Cerebral index	Within-group differences		
	Affected/non-domH	Unaffected/domH		Affected/non-domH vs. unaffected/domH	Affected/non-domH vs. cerebral index	Affected/domH vs. cerebral index
Healthy	2.08 ± 0.70	2.11 ± 0.67	2.09 ± 0.71	—	—	—
Poststroke patients	5.39 ± 2.44	4.85 ± 2.09	5.07 ± 2.18	*t* = −2.38; *p* = 0.02	*t* = 2.51; *p* = 0.01	*t* = −2.04; *p* = 0.04
Mild/moderate	4.67 ± 1.90	4.49 ± 1.78	4.54 ± 1.74	—	—	—
Severe	6.21 ± 2.7	5.27 ± 2.37	5.66 ± 2.49	*t* = −2.35; *p* = 0.02	*t* = 2.33; *p* = 0.03	*t* = −2.17; *p* = 0.04

non-domH: nondominant hemisphere; domH: dominant hemisphere. Data are mean ± SD. Significant post hoc test values for within-group differences are shown.

The article "Intrahemispheric EEG: A New Perspective for Quantitative EEG Assessment in Poststroke Individuals" was published in 2021. Journal: Neural Plast.

## Data Availability

The data that support the findings of this study are available from the corresponding author (DP) upon reasonable request.
